This article has been retracted.

# *Allium cepa* L. and Quercetin Inhibit RANKL/*Porphyromonas gingivalis* LPS-Induced Osteoclastogenesis by Downregulating NF-*κ*B Signaling Pathway

**DOI:** 10.1155/2015/704781

**Published:** 2015-07-26

**Authors:** Tatiane Oliveira, Camila A. Figueiredo, Carlos Brito, Alexander Stavroullakis, Ana Carolina Ferreira, Getulio Nogueira-Filho, Anuradha Prakki

**Affiliations:** ^1^Departamento de Bio-Regulação, Instituto de Ciências da Saúde, Universidade Federal da Bahia, 40.110-100 Salvador, BA, Brazil; ^2^Department of Clinical Sciences, University of Toronto, Restorative, Toronto, ON, Canada M5G 1G6

## Abstract

*Objectives*. We evaluated the *in vitro* modulatory effects of *Allium cepa* L. extract (*AcE*) and quercetin (Qt) on osteoclastogenesis under inflammatory conditions (LPS-induced). *Methods*. RAW 264.7 cells were differentiated with 30 ng/mL of RANKL, costimulated with *Pg*LPS (1 *µ*g/mL), and treated with *AcE* (50–1000 *µ*g/mL) or Qt (1.25, 2.5, or 5 *µ*M). Cell viability was determined by alamarBlue and protein assays. Nuclei morphology was analysed by DAPI staining. TRAP assays were performed as follows: p-nitrophenyl phosphate was used to determine the acid phosphatase activity of the osteoclasts and TRAP staining was used to evaluate the number and size of TRAP-positive multinucleated osteoclast cells. Von Kossa staining was used to measure osteoclast resorptive activity. Cytokine levels were measured on osteoclast precursor cell culture supernatants. Using western blot analysis, p-I*κ*B*α* and I*κ*B*α* degradation, inhibitor of NF-kappaB, were evaluated. *Results*. Both *AcE* and Qt did not affect cell viability and significantly reduced osteoclastogenesis compared to control. We observed lower production of IL-6 and IL-1*α* and an increased production of IL-3 and IL-4. *AcE* and Qt downregulated NF-*κ*B pathway. *Conclusion*. *AcE* and Qt may be inhibitors of osteoclastogenesis under inflammatory conditions (LPS-induced) via attenuation of RANKL/*Pg*LPS-induced NF-*κ*B activation.

## 1. Introduction

Normal inflammatory responses are tightly controlled and self-limiting. Chronic inflammation, however, can lead to an abnormal increase in osteoclastic bone resorption and excessive bone destruction as observed in osteoporosis, rheumatoid arthritis, and periodontal disease (PD) [1–3]. Osteoclasts are multinucleated cells which are capable of degrading bone matrix and play an important role in physiological bone development and remodeling [4]. Studies have demonstrated that the etiology of PD derives from periodontal pathogenic bacteria, such as* Porphyromonas gingivalis* [5]. The LPS, a major constituent of the cell wall of such Gram-negative bacteria, has long been recognized as a key factor implicated in the development of chronic periodontitis [6]. It is the host immune response to these oral microorganisms that leads to the destruction of periodontal bone tissues by production of nuclear factor kappa B ligand (RANKL) that is expressed on T lymphocytes in human periodontal disease [7].

The stimulation of mononuclear osteoclast progenitors by macrophage colony-stimulating factor (M-CSF) and the activation of nuclear factor-*κ*B by RANKL which induce their differentiation along the osteoclastic lineage and their fusion into mature, multinucleated osteoclasts are crucial for osteoclastogenesis [8].

A previous study has revealed that lipopolysaccharides are also involved in osteoclastogenesis via the stimulation of osteoblasts to produce an excess of RANKL [9]. Additionally, several proinflammatory cytokines have been identified as direct or indirect stimulators of osteoclast differentiation, survival, and activity. Cytokines modulate inflammatory responses and activate different intracellular pathways to initiate osteoclast differentiation [10]. These include interleukin-1 (IL-1), tumor necrosis factor-alpha (TNF) [11], interferon-gamma (IFNg), interleukin-6 (IL-6), and, very importantly, RANKL that directly induces osteoclastogenesis [12]. Conversely, other cytokines such as IFN-*γ*, IL-3, and IL-4 can act as osteoclastogenic inhibitors [13].

Recently, the importance of using natural products has increased, as has the interest in discovering safe and efficient new drugs to treat inflammatory conditions [14]. Studies have investigated the use of natural products in the treatment of various inflammatory diseases such as asthma [15], ulcerative colitis [16], Crohn's disease [17], and bone loss in inflammatory conditions such as periodontitis [9]. Of these products, flavonoids contained in fruits and vegetables have been found to be very active as anti-inflammatory agents [18]. The major flavonoid found in* Allium cepa* L. (onion) is quercetin (Qt) which exhibits many pharmacological properties such as anti-inflammatory and antioxidant effects [19–21]. Qt is also a potent inhibitor of* in vitro* osteoclastic differentiation [22].* Allium cepa* L. extract (*AcE*) has also been studied to treat inflammatory conditions such as asthma [23], ovariectomy-induced bone resorption in rats [24], and the inhibition of RANKL-induced ERK, p38, and NF-*κ*B activation in osteoclasts precursor cells in rats [25]. The modulation of osteoclast formation and function is a promising strategy for the treatment of bone-destructive and inflammatory diseases [3]. Thus, this study was designed to investigate whether* Allium cepa *L. and quercetin exert effects on osteoclasts and their precursors under normal and LPS-induced inflammatory conditions. Osteoclastogenesis and osteoclast activity were observed through modulation of inflammatory mediators and through measurement of the expression of IkappaB-*α* which is an inhibitor of cytoplasmic NF-kappaB in RANKL/*Pg*LPS-induced osteoclast precursor cells.

## 2. Material and Methods

### 2.1. Chemicals and Reagents

Murine macrophage cells (RAW 264.7) were obtained from the American Type Culture Collection (ATCC Accession number TIB-71). Dulbecco's modified Eagle's medium (DMEM), Minimum Essential Medium Eagle (*α*-MEM), and Fetal Bovine Serum (FBS) were purchased from Invitrogen-Gibco (Carlsbad, CA, USA). The mouse IL-3 (Cat number 432102, Lot: B154176), IL-4 (Cat number 431102, Lot: B156652), IL-6 (Cat number 431305, Lot: B165924), IL-1*α* (Cat number 433402, Lot: B171801), TNF (Cat number 430902, Lot: B170648), and enzyme-linked immunosorbent assay (ELISA) kit were purchased from BioLegend's ELISA MAX (San Diego, CA, USA). LPS derived from* P. gingivalis *(*Pg*) was purchased from Cedarlane (Ontario, Canada). For cells viability assay, alamarBlue was purchased from Invitrogen (Cat number DAL1025) (Grand Island, NY, USA) and protein concentrations were determined by Pierce BCA from Thermo Scientific (Cat number 23225) (Rockford, IL, USA). Mouse-derived RANKL, dimethyl sulfoxide (DMSO) ≥99.5%, penicillin G-streptomycin, acid phosphatase kits for tartrate-resistant acid phosphatase (TRAP) staining, 4,6-diamidino-2-phenylindole (DAPI) for DAPI staining, quercetin 98% (2-(3,4-dihydroxyphenyl)-3,5,7-trihydroxy-4H-1-benzopyran-4-one,3,3′,4′,5,6-entahydroxyflavone), and the other chemicals were purchased from Sigma Aldrich (St. Louis, MO, USA).

### 2.2. *Allium cepa* L. extract (*AcE*)

*Allium cepa* L. extract was obtained as previously described [26]. Briefly, samples were peeled, cut, and successively extracted three times with methyl alcohol (CH_3_OH) 99.8% during 7 days. After filtering, the extract was concentrated by evaporation under reduced pressure using a rotary evaporator. After the solvent was removed, the* AcE* was dried in the oven and kept in −20°C during the experimental phase. The standardization of* Allium cepa *L. extract was performed by High Performance Liquid Chromatography (HPLC). The calculated average percentage of Qt in the* AcE* extract was 2.5% [27]. Different concentrations of* AcE* (100, 500, or 1000 *μ*g/mL) and Qt (1.25, 2.5, or 5 *μ*M) were solubilized at noncytotoxic concentrations of DMSO (0.05%) and were tested. The concentrations of* AcE* were selected based on a previous* in vitro* study that demonstrated no toxicity effect of* AcE* in same concentrations towards* Porphyromonas gingivalis* LPS and* Escherichia coli* LPS-induced osteoclast precursor cells [26].

### 2.3. Cell Culture

RAW 264.7 mouse monocyte macrophage cell lines used as an osteoclast precursor were seeded (5 × 10^6^ cells/well) in culture flasks (75 mL BD Falcon, Franklin Lakes, NJ, USA) as previously described [28]. The cells were maintained in DMEM containing 10% Fetal Bovine Serum (FBS), 100 U/L penicillin G, and 100 mg/L streptomycin at 37°C with 5% CO_2_. The medium was changed every 2 days.

### 2.4. Osteoclast Differentiation

Initial experiments were designed to evaluate the effects of test compounds on osteoclastogenesis and osteoclast activity under inflammatory conditions. For these experiments, after 3 days of cell growth, the RAW 264.7 cells were plated in 96-well plates at a density of 5 × 10^3^ cells/well containing *α*-MEM medium, 10% FBS, 2 mM L-glutamine, and 100 *μ*g/mL penicillin/streptomycin. After overnight incubation, culture medium was replaced and the cells were stimulated with vehicle (untreated control) or 30 ng/mL of RANKL and 1 *μ*g/mL* Pg*LPS, in order to induce cell differentiation and infection in a simultaneous manner. At this time, the tested concentrations of* AcE* (100, 500, or 1000 *μ*g/mL), Qt (1.25, 2.5, or 5 *μ*M) were added to the wells for 5 days with change of medium on day 3.

### 2.5. Cell Viability Assays

#### 2.5.1. Image Analysis and Cell Count by DAPI Staining

To determine the noncytotoxic concentrations of* AcE* or Qt on the RAW 264.7 osteoclast precursor cell line, cells were grown in 96-well plates in the presence and absence of* AcE* (100, 500, or 1000 *μ*g/mL) or Qt (1.25, 2.5, or 5 *μ*M) and vehicle with DMSO 0.05% (cell) during 5 days. DMSO (50%) was used for positive control. Fluorescence images stained by 4,6-diamidino-2-phenylindole (DAPI) (*n* = 3, *N* = 3) were performed to evaluate the morphology and cell counts as previously described [26]. Cells were stained with 4,6-diamidino-2-phenylindole (DAPI), and those with fragmented or condensed nuclei were defined as apoptotic cells [29]. Five visual images were taken using fluorescent microscopy (Cytation 3, Biotek, USA) and each sample was analyzed using Gen5 software (Biotek, USA).

#### 2.5.2. Resazurin Reduction and Protein Assays

Resazurin reduction assay (alamarBlue) (*n* = 3, *N* = 3) was performed to analyze viable cells with active metabolism on osteoclastogenesis under inflammatory conditions as previously described [26, 30]. For these experiments, RAW 264.7 macrophages were cultured in the presence of vehicle or RANKL and LPS and in the presence and absence of* AcE* (100, 500, or 1000 *μ*g/mL) or Qt (1.25, 2.5, or 5 *μ*M) for 5 days. The cultures were placed in medium containing 10% of alamarBlue. After 4 h of incubation, 100 *μ*L of the medium was transferred to the wells of a 96-well plate and the optical density (OD) was measured using a BioRad ELISA 3550 plate reader at wavelengths of 570 nm and 600 nm. The percentage of cells showing cytotoxicity relative to the control group (Ctrl) was determined. A greater percentage reduction of alamarBlue reflects greater cell proliferation. Protein assay was used to confirm the effect of* AcE* on cell viability. The protein concentration in all tested samples was compared to a protein standard. Cell lysis was carried out as listed in Kartner et al. [30]. Cells were briefly washed with PBS and lysed with protein lysis buffer (90 mM trisodium citrate, 10 mM NaCl, 0.1% Triton X-100, pH 4.8). The OD was measured using a BioRad ELISA 3550 plate reader at a wavelength of 562 nm which provided the formula to calculate the protein levels.

### 2.6. Tartrate-Resistant Acid Phosphatase (TRAP) Assays

To examine the inhibitory effect of* AcE* and Qt on RANKL/*Pg*LPS-induced osteoclastogenesis in RAW 264.7, quantitative and qualitative measurements of TRAP (*n* = 3, *N* = 3) were obtained using two methods previously described [31]. Osteoclast formation was measured by quantifying cells that were positively stained by TRAP. The number of TRAP+ multinucleated osteoclasts per well was determined, small osteoclasts (2–5 nuclei) and large ones (+10 nuclei), using light microscopy. Digital images of TRAP+ cells were taken under brightfield microscopy using a Leica DM IRE2 microscope with OpenLAB software (Leica Microsystems). Image analysis was performed with NIH ImageJ 1.46r software. Additionally, the total soluble TRAP activity was determined from cells permeabilized by means of an acidic detergent buffer, in order to measure the acid phosphatase activity of the osteoclasts using a microplate reader (405 nm). The amount of* p*-nitrophenol released indicates the degree of cell differentiation.

### 2.7. Hydroxylapatite Resorption Assay (Von Kossa Staining)

Mineral accumulation was visualized by histochemical Von Kossa staining for calcium phosphate. Resorption assays on Corning Osteo Assay surface 24-well plates (*n* = 3, *N* = 3) (Cat number 3987), Corning Life Sciences, Corning, NY, USA, were performed as per Kartner et al. [30]. Briefly, RAW 264.7 cells were differentiated into osteoclasts and allowed to attach to plates for 2 h at 37°C with 100 mL of medium containing 30 ng/mL RANKL. On day 5, the RAW cells were transferred to Osteo Assay plates and tested with* AcE* (100, 500, and 1000 *μ*g/mL) or Qt (1.25, 2.5, or 5 *μ*M) concentrations. After 24 h, cells were stripped from plates with 500 mL of 1.2% sodium hypochlorite for 5 min. The plates were then aspirated, washed thoroughly with water, and air-dried prior to staining. Modified Von Kossa staining was used to increase the contrast of the Osteo Assay. Darkfield microscopy showed individual or multiple resorption pits at 40x magnification.

### 2.8. Cytokine Assay

Cytokine levels were measured in the supernatants collected from RAW 264.7 cells in the presence and absence of RANKL (30 ng/mL)/*Pg*LPS (1 *μ*g/mL) and* AcE* (100, 500, or 1000 *μ*g/mL) or Qt (1.25, 2.5, or 5 *μ*M) with a commercially available ELISA kit (*n* = 3, *N* = 3). The secretions of interleukin-6 (IL-6), IL-3, IL-4, TNF, and IL-1*α* were measured in the supernatants collected during osteoclast differentiation (after 24 h, 3 days, and 5 days) and after 24 h on the Osteo Assay surface plates to measure the osteoclast activity. Briefly, cell culture supernatants were collected and centrifuged to remove cellular debris. Samples were incubated with polyclonal antibodies specific for mouse (IL-6, IL-3, IL-4, TNF, and IL-1*α*) and then enzyme-linked substrate. The intensity of the color detected at 450 nm (background wavelength 570 nm) was measured after the addition of a substrate solution, and cytokine concentrations were calculated from the standard curve prepared by diluting the standard solution provided in the kit.

### 2.9. Western Blot Analysis

RAW 264.7 cells were seeded for 2 hours and pretreated in the presence and absence of the optimal concentration of* AcE* (1000 *μ*g/mL) or Qt (5 *μ*M) along with an untreated control for 1 hour. Afterwards, cells were stimulated with RANKL and* Pg*LPS within 30 minutes as listed in Xie et al. [32]. The cells treated with indicated reagents were lysed in RIPA buffer with protease and phosphatase inhibitors (Cell Signaling, Danvers, MA). Cell lyses were centrifuged at 13,000 rpm for 20 minutes to remove cell debris. Equal transfer of proteins was confirmed by BioRad protein assay reagent. The lysate (10 *μ*g protein/lane) was separated by sodium dodecyl sulfate polyacrylamide gel electrophoresis and transferred to a nitrocellulose membrane. After transfer, the membrane was blocked for 2 hours with 5% bovine serum albumin/phosphate buffered saline containing 0.05% Tween-20 and then probed with antibodies against I*κ*B*α* (Santa Cruz Biotechnology, mouse monoclonal IgG_1_, Lot number I1212, Cat number sc-1643), p-I*κ*B*α* (rabbit polyclonal IgG, Lot number A0413, Cat number sc-7977), and *β*-actin (Cell Signaling, Rabbit mAb, Lot number 11, Cat number 4970P). The dilution ratio was 1 : 1,000. After three washes, the membranes were subsequently incubated for 2 hours with anti-I*κ*B*α* (Santa Cruz Biotechnology, Goat anti-mouse IgG-HRP, Lot number Lo312, HRP conjugated Cat number sc-2005), anti-p-I*κ*B*α* (Goat anti-rabbit IgG-HRP, Lot number A0713, HRP conjugated Cat number sc-2004), and anti-*β*-actin (Goat anti-rabbit IgG-HRP, Lot number A0713, HRP conjugated Cat number sc-2004). For both anti-mouse and anti- rabbit, the dilution ratio was 1 : 5,000. The antigens were detected using enhanced chemiluminescence (ECL) reagents (GE Healthcare, Piscataway, NJ) according to the manufacturer's instructions. The bands were analyzed using MyECL Imager (Thermo Scientific, Rockford, IL, USA) (*N* = 3).

### 2.10. Statistical Analysis

For each assay, statistical significance was determined by ANOVA followed by Tukey's pairwise comparisons to detect specific differences between tested groups and control (*α* = 0.05). Statistical analyses were performed using GraphPad Prism (GraphPad Software Inc., San Diego, CA, USA). Each experiment was carried out in triplicate and repeated at least three times.

## 3. Results

### 3.1. *AcE* and Qt Do Not Induce Cell Proliferation and Apoptosis in RAW 264.7 Cells

According to the cell viability assays, the tested concentrations of* AcE* or Qt were not toxic to this specific cell line. RAW cells were cultured in the presence of* AcE* (100, 500, or 1000 *μ*g/mL) or Qt (1.25, 2.5, or 5 *μ*M) during 5 days.* AcE* and Qt did not negatively affect cell viability when compared with negative control (cell) as investigated by DAPI staining as shown in Figures 1(a) and 1(b).

Additionally, resazurin reduction was performed to confirm that* AcE* and Qt had no significant toxic effects in RANKL/*Pg*LPS-induced osteoclastogenesis. Concomitant total protein assay confirmed that RAW 264.7 RANKL/*Pg*LPS-induced cell viability was unaffected at the* AcE *and Qt working concentrations as shown in Figures 2(a) and 2(b).

### 3.2. *AcE* and Qt Affected RANKL/*Pg*LPS-Induced RAW 264.7 Cells during Osteoclastogenesis

To determine the effect of* AcE* and Qt on osteoclast differentiation under RANKL/*Pg*LPS-stimulation, using the RAW 264.7 cell system, the number of TRAP+ multinucleated cells was determined per well. In the absence of LPS, RANKL,* AcE,* and Qt, no osteoclasts are seen (Figure 3(a)(A)). The presence of both LPS and RANKL significantly increased the differentiation of osteoclasts from RAW 264.7 cells (Figure 3(a)(B)). All three concentrations of* AcE* (100, 500, or 1000 *μ*g/mL) and Qt (1.25, 2.5, or 5 *μ*M) inhibited RANKL/*Pg*LPS-induced osteoclast formation (*p* < 0.001) (Figure 3(a)(C)–(H)). When compared to control, a decrease in small osteoclasts (*p* < 0.01) was observed in the highest concentration of* AcE* (1000 *μ*g/mL) and in two concentrations of Qt (2.5, 5 *μ*M) (*p* < 0.05) (Figures 3(b) and 3(c)). In addition, a significant decrease in the amount of* p*-nitrophenol released was observed with all* AcE* and Qt concentrations tested when compared to the control (Figure 3(d)).

### 3.3. *AcE* and Qt Decrease Osteoclast Resorptive Activity

Figure 4(a) shows the raw and contrast images of Osteo Assay surface partially resorbed by RANKL/*Pg*LPS-induced osteoclast (Ctrl) compared to the untreated control (cell).  Figure 4(b) shows quantification of inhibition by* AcE* and Qt of Osteo Assay surface resorption by RANKL/*Pg*LPS-induced osteoclast as indicated. Treatment with the three concentrations of* AcE* and Qt significantly reduced the effects of RANKL/*Pg*LPS on osteoclast activity. Thus, to assess more precisely how resorption pit morphology was affected by* AcE* or Qt, pit areas were quantified and calculated using ImageJ 1.46r. These data are represented in graph format (Figure 4(b)). All* AcE* and Qt concentrations significantly decreased overall resorption pit area (*p* < 0.001).

### 3.4. *AcE* and Qt Affect Cytokine Production during Osteoclastogenesis and Osteoclast Activity

The effect of* AcE* and Qt on the production of inflammatory mediators by RANKL/*Pg*LPS-induced osteoclast was investigated by measuring the levels of cytokines during osteoclastogenesis and osteoclast activity. During osteoclast formation in day 5, IL-1*α* secretion was decreased on* AcE* at 100 *μ*g/mL, 500 *μ*g/mL, and 1000 *μ*g/mL (*p* < 0.001) and by Qt 2.5 and 5 *μ*M (*p* < 0.001). IL-6 secretion also was decreased by* AcE* at 500 *μ*g/mL and 1000 *μ*g/mL (*p* < 0.01), and also all concentrations of Qt tested compared to control. IL-3 secretion was increased by* AcE* 1000 *μ*g/mL (*p* < 0.01) and by Qt (*p* < 0.05), and IL-4 secretion was increased by* AcE* 1000 *μ*g/mL (*p* < 0.05). The cytokine production was not affected by* AcE* or Qt during osteoclastogenesis at 24 h or 3 days. After 24 h of osteoclast activity, IL-1*α* secretion was decreased by* AcE* 100 *μ*g/mL and 500 *μ*g/mL (*p* < 0.01)* AcE* at 1000 *μ*g/mL (*p* < 0.001) and by Qt 5 *μ*M (*p* < 0.01). IL-6 secretion was decreased by* AcE* at 1000 *μ*g/mL (*p* < 0.01) and by Qt 5 *μ*M (*p* < 0.05), while TNF secretion was not modulated by* AcE* or Qt when compared to control (RANKL.LPS) (Table 1).

### 3.5. *AcE* and Qt Inhibit RANKL/*Pg*LPS-Induced NF-*κ*B Activation

The molecular mechanisms that underlie the role of* AcE* and Qt in the process of osteoclast differentiation were determined by examining the effect of these compounds on the phosphorylation and degradation of I*κ*B*α*. RANKL/*Pg*LPS stimulation induced within 30 min (Figure 5) the phosphorylation of I*κ*B*α*.* AcE* and Qt decreased the levels of I*κ*B*α* phosphorylation, whereas the nonphosphorylated forms of I*κ*B*α*, inhibitor of cytoplasmic NF-kappaB (*p* < 0.001), were not affected. In addition,* AcE* and Qt blocked I*κ*B*α* degradation (*p* < 0.001).

## 4. Discussion

The etiological roles of periodontal bacteria, such as* P. gingivalis*, in the onset and progression of PD, are well documented, as well as the engagement of periodontal bacteria in RANKL-mediated alveolar bone resorption [9]. Natural compounds have been proposed as one of the groups of bioactive components in plant-based foods responsible for the beneficial effects on inflammatory disease [32] and bone metabolism [28].* Allium cepa* L. has been studied to treat inflammatory conditions [23] and bone resorption [24].* AcE* also inhibits activation of osteoclast precursor cells [25]. In the course of investigations into the biologically active metabolites of* Allium cepa* L., quercetin was isolated as a major constituent of this species [21, 22]. Previous studies have already demonstrated the effects of* Allium cepa* L. and quercetin in RANKL-induced osteoclastogenesis; however, this study is the first to demonstrate how these compounds influence osteoclast precursors and their differentiation into mature, bone-resorbing osteoclasts under RANKL/*Pg*LPS-induced differentiation and inflammation.

Under conditions of chronic inflammation, RANKL-mediated osteoclastogenesis is enhanced by oxidative stress and proinflammatory molecules including tumor necrosis factor (TNF) [33], interleukin- (IL-) 1, IL-6 [13], nitric oxide (NO) [34], and lipopolysaccharide (LPS) [32]. In this study, we investigated the direct effects of these compounds on osteoclast precursors and mature osteoclasts in the presence of RANKL under inflammatory conditions through* Pg*LPS induction, and we found that both* AcE* and Qt were able to suppress osteoclast differentiation and activity even in the presence of RANKL/*Pg*LPS in RAW 264.7 cells. These effects on osteoclastogenesis and resorption activity occurred in parallel with the modulation of inflammatory mediators and downregulation of NF-*κ*B. In patients with inflammatory diseases, bone loss or osteolysis can be a result of either excessive bone resorption or decreased bone formation, or a combination of these processes [2]. In this study, we demonstrated that* AcE* and Qt modulate the inflammatory process and osteoclast activity. However, it has been previously described that aqueous* Allium cepa* L. extract did not directly affect the cell proliferation and differentiation of human osteoblasts, which are responsible for bone formation [25]. Moreover, other natural products, such as polyphenols from dried plum, have been shown to inhibit osteoclastogenesis, under inflammatory conditions induced by lipopolysaccharide (LPS), leading to a decrease in osteoclast activity, by downregulating NFATc1 and inflammatory mediators [28]. Previous studies showed the effects of AcE extract or Qt on osteoclast formation and activities* in vivo* [24, 35] and* in vitro *[25]. In the present study, the expression of NF-kappaB's inhibitory protein and IkappaB-alpha was measured and it was verified that the inhibition of osteoclastogenesis caused by AcE extract or Qt can be partly attributed to the maintenance of IkappaB-alpha, a cytoplasmic trapper or inhibitor of NF-kappaB.

It has been established that IL-1*α*, IL-6, and TNF directly or indirectly promote osteoclastogenesis, whereas IL-3, IL-4, alone or in synergy with other cytokines, inhibit osteoclasts formation [13, 28]. In this study, we demonstrated that the evaluated compounds decreased the secretion of IL-1*α* and IL-6 during osteoclast formation and activity when compared to the positive controls. However, a reduction in the secretion of TNF was also shown to occur. These results suggest that* AcE* and Qt may be relevant in the attempt to inhibit the secretion of cytokines that promote inflammation and bone loss. Moreover, it was demonstrated that* AcE* and Qt stimulated the secretion of IL-3 and IL-4, inhibiting osteoclastogenesis.

In addition to the effect on inflammatory mediators,* AcE* and Qt downregulated NF-*κ*B on osteoclastogenesis under inflammatory conditions (*Pg*LPS-induced).

Lipopolysaccharide stimulation elicits a cascade leading to the activation of NF-*κ*B that leads to the production of inflammatory cytokines. Several mechanisms underlying the inhibition of LPS-induced inflammatory cytokine production by flavonoids have been investigated, of which the blocking of NF-*κ*B pathways has been proposed as the one major mechanism. Thus, inhibition of the LPS-induced signal transduction cascades has been proposed as a promising target for the treatment of inflammation [32].

The activation pathway of NF-*κ*B by most inflammatory agents requires both phosphorylation and degradation of the inhibitory subunit I*κ*B*α* [25, 32]. In this study, pretreatment with* AcE* or quercetin attenuated the RANKL/*Pg*LPS-induced of I*κ*B-*α* degradation and I*κ*B*α* phosphorylation, which may partly explain its strong inhibitory effect in attenuating NF-*κ*B activation and consequently the cytokine production in our* in vitro *model.

It is reasonable to argue at this time that the effects on osteoclastogenesis and osteoclast activity reported here are the result of the action of* AcE* as a whole and not only of quercetin. This study demonstrated that the inhibitory activity of quercetin tested is similar to the effect produced by the extract, but the extract tested is composed only by 2.5% of quercetin [27].

Thus, further studies are needed to investigate the anti-inflammatory potential of other specific compounds of* Allium cepa* L. in the effect of RANKL/*Pg*LPS-induced osteoclastogenesis and osteoclast activity. In conclusion,* Allium cepa* L. extract and quercetin may be considered inhibitors of osteoclastogenesis and osteoclast activity under inflammatory conditions (LPS-induced). This is likely to happen via attenuation of NF-*κ*B activation signaling pathway in osteoclasts precursor cells. Further studies are needed in order to explore long-term effect of* AcE* and Qt exposure to support the use of both drugs in the treatment of diseases involving pathological bone loss including periodontitis.

## Figures and Tables

**Figure 1:** *AcE* and Qt do not induce cell proliferation and apoptosis in RAW 264.7 cells. RAW cells were cultured for 5 days in the presence of various concentrations of* AcE* and Qt. (a) Morphology of apoptotic cell nuclei was observed: (A) cell, (B)* AcE* 100 *μ*g/mL, (C)* AcE* 500 *μ*g/mL, (D)* AcE* 1000 *μ*g/mL, (E) Qt 1.25 *μ*M, (F) Qt 2.5 *μ*M, (G) Qt 5 *μ*M, and (H) DMSO. (b) Cell count by DAPI staining using a fluorescence microscope. There was no significant difference between negative control (cell) and cells in all concentrations tested. There was significant difference between positive control (DMSO) and cells in all concentrations tested (^*∗∗∗*^ *p* < 0.001) using ANOVA and Tukey's post hoc test. Results were expressed in mean ± SD of three independent experiments.

**Figure 2:** *AcE* and Qt are not toxic to RANKL/*Pg*LPS-induced RAW 264.7 cell. Cells were cultured in the presence of* Pg*LPS, RANKL, and* AcE* or Qt. Negative control (Ctrl) cells were not exposed to* AcE* or Qt. After 5 days of continuous exposure, cell viability was assessed using alamarBlue assay (a) and total protein levels were assessed using protein assays (b). There was no significant difference between control (Ctrl) and cells in all concentrations tested, ANOVA-Tukey test. Results were expressed in mean ± SD of three independent experiments.

**Figure 3:** RANKL*/Pg*LPS-induced RAW 264.7 cells were affected by* AcE* or Qt during osteoclastogenesis. (a) TRAP staining by brightfield microscope showed differentiated osteoclasts in the presence of* AcE* or Qt after 5 days. The arrows show decreased size of osteoclasts; TRAP-stained, fixed cultures were for number of nuclei per cell in two different groups: (b) 2–5 small and (c) +10 large nuclei per cell. (d) The acid phosphatase activity of the osteoclasts was decreased in all* AcE* and Qt concentrations tested: ^*∗*^ *p* < 0.05, ^*∗∗*^ *p* < 0.01, and ^*∗∗∗*^ *p* < 0.001 when compared with Ctrl group according to the ANOVA and Tukey tests. Results were expressed in mean ± SD of three independent experiments.

**Figure 4:** *AcE* and Qt decrease osteoclast resorptive activity in all concentrations tested. (a) RANKL-induced RAW 264.7 cells were differentiated into osteoclasts for 5 days and transferred to Corning Osteo Assay plates. The mature cells were tested in the presence of PgLPS, RANKL, and* AcE* or Qt for 24 h and untreated group (Ctrl) was not exposed to* AcE* or Qt. Von Kossa stain was performed on all samples tested, and the plates were air-dried and imaged using digital brightfield photomicrography. Images shown are ImageJ software processed for quantification. The images show unresorbed areas appear black, and areas of resorption are white. (b) Quantification of (a): ^*∗∗∗*^ *p* < 0.001, ANOVA-Tukey test. Results were expressed in mean ± SD of three independent experiments.

**Figure 5:** *AcE* (a) and Qt (b) modulate* Pg* RANKL/*Pg*LPS-induced I*κ*B degradation in RAW 264.7 macrophages. Cell lysates were analyzed by immunoblotting by reacting with antibodies anti-I*κ*B*α* and I*κ*B*α*-p. *β*-actin served as the control for the protein assay. Blots were performed three times, and averaged expression levels were normalized to *β*-actin as indicated above each blot, denoting statistical significance according to ANOVA and Tukey's post hoc test with ^*∗∗∗*^ *p* < 0.001.

**Table 1:** *AcE* and Qt affect cytokine production during osteoclastogenesis and osteoclast activity. The supernatant was collected and IL-1*α*, IL-6, TNF, IL-3, and IL-4 levels were measured during osteoclastogenesis (24 hours, 3 days, and 5 days) and osteoclast activity (24 hours).

Cytokine (pg/mL)	Control		Test compounds					
			*AcE*			Qt		
	Cell	Ctrl	[100 *µ*g/mL]	[500 *µ*g/mL]	[1000 *µ*g/mL]	[1,25 *µ*M]	[2,5 *µ*M]	[5 *µ*M]
Osteoclastogenesis								

Time, 24 hours								
IL-1*α*	31.77	40.22	39.54	36.02	36.70	33.76	34.21	32.85
IL-6	68.77	90.01	84.88	84.42	82.40	81.93	87.37	84.88
TNF	230	299	228	242	281	247	264	264
IL-3	64.88	59.93	59.73	58.72	62.86	58.01	57.71	58.11
IL-4	66.84	58.69	60.32	60.48	60.65	59.34	57.55	62.44

Time, 3 days								
IL-1*α*	21.77	39.54^#^	39.31	37.38	36.93	37.95	41.01	41.92
IL-6	43.35	72.29^###^	69.49	66.93	61.22	62.22	69.71	71.59
TNF	70	174^###^	153	145	167	161	159	172
IL-3	51.24	43.23	40.43	47.30	53.53	52.35	50.73	50.33
IL-4	58.20	52.66	54.13	52.99	54.62	60.97	58.86	59.34

Time, 5 days								
IL-1*α*	168	221^###^	156^*∗∗∗*^	97^*∗∗∗*^	110^*∗∗∗*^	200	144^*∗∗∗*^	135^*∗∗∗*^
IL-6	66.09	98.42^###^	80.08^*∗∗∗*^	81.32^*∗∗∗*^	82.25^*∗∗∗*^	78.06^*∗∗∗*^	78.37^*∗∗∗*^	79.30^*∗∗∗*^
TNF	34.76	76.10^###^	75	70.01	64.40	64.55	65.80	63.62
IL-3	50.13	42.65^##^	40.43	44.27	51.14^*∗∗*^	30.7	40.73	49.22^*∗*^
IL-4	62.24	50.38^#^	51	54.54	61.87^*∗*^	50.87	54.66	49.65

Osteoclast activity								

Time, 24 hours								
IL-1*α*	88.53	126.8^#^	82.27^*∗*^	75.46^*∗*^	69.51^*∗∗*^	129.3	109.7	81.72^*∗∗*^
IL-6	29.74	70.07^#^	50.61	56.67	25.08^*∗*^	60.75	55.85	31.14^*∗*^
TNF	67.36	131.9^#^	99.33	94.89	99.33	95.75	92.16	105.1

The following denotes statistical significance: ^#^ *p* < 0.05, ^##^ *p* < 0.01, and ^###^ *p* < 0.001 when compared with cell group and ^*∗*^ *p* < 0.05, ^*∗∗*^ *p* < 0.01, and ^*∗∗∗*^ *p* < 0.001 when compared with Ctrl group, verified by ANOVA-Tukey test. Results were expressed in mean ± SD of three independent experiments.
